The article "“I Could Really Use This”: Occupational Therapy Students' Perceptions of Learning to Coach" was published in 2022. Journal: Occup Ther Int.

# “I Could Really Use This”: Occupational Therapy Students' Perceptions of Learning to Coach

**DOI:** 10.1155/2022/2266326

**Published:** 2022-10-13

**Authors:** Marie-Christine Potvin, Erin K. West, Alexis N. Morales, Katherine S. Sailor, Natalie Coronado

**Affiliations:** Department of Occupational Therapy, College of Rehabilitation Sciences, Thomas Jefferson University, 901 Walnut Street, 6th Floor, Philadelphia, PA 19107, USA

## Abstract

Coaching, an evidence-based approach in other fields, is relatively novel within occupational therapy (OT) and is not yet widely taught in OT programs. In recent studies, experienced occupational therapists have reported that coaching added value to their practice, but OT students' perspectives are missing from the literature. This phenomenological study explored OT students' (*n* = 14) perceptions of the value of learning to coach while in fieldwork. Three themes emerged from the inductive qualitative analysis: *Coaching Requires a Mindset Shift*, *Change is a Journey*, and *Impact on Clients*. Occupational therapy students perceived that coaching required a different way of thinking and reimagining their role, saw the value of learning to coach in the clients' outcomes, and recognized the potential for their future practice regardless of settings. The study findings suggest that incorporating coaching skills into OT education could be beneficial to students when they enter the profession.

## 1. Introduction

Coaching is an evidence-based approach used in various professions to help clients reach their goals [1]. The use of coaching within occupational therapy (OT) is relatively novel; the earliest study was published in 2010 [2]. So far, studies of OT-led coaching have all had positive outcomes regardless of populations including cerebral palsy, stroke, and autism spectrum disorder [2–8]; Mulcahey et al., [9]. In-depth training in coaching is needed before OT practitioners can effectively integrate coaching into their practice [6, 10]. Coaching requires a unique skill set that is not taught to most OT students in their entry-level curriculum [11]. The perspective of licensed occupational therapists who received training in coaching has been investigated [6, 12], but there is no research on the OT student perspective of learning this approach within entry-level OT education.

### 1.1. What Is Coaching?

The International Coaching Federation (ICF), a premier coaching credentialling organization, defines coaching as partnering with clients in a thought-provoking and creative process that inspires them to maximize their personal and professional potential [13]. Over the last 25 years, the ICF has developed and updated coaching competencies that specify the behaviors and skills of coaches (e.g., listen actively, evoke awareness, and facilitate client's growth), with the partnership between coach and client being central [14]. Many approaches labelled as “coaching” in the literature would not meet the ICF definition, as they include strategies such as teaching, modeling, scaffolding, and guiding [15]; ICF-style coaching does not include such strategies except in rare occasions, at clients' request. The ICF coaching competencies have been operationalized in a variety of coaching models (e.g., executive coaching, solution-focused coaching, positive psychology coaching, and academic coaching) used by professional coaches and others who adopt coaching as part of their practice [1, 12, 16–18]. Coaching approaches aligned with ICF definitions and competencies emerged within OT research in the early 2010s [2, 9, 19–21].

The article "“I Could Really Use This”: Occupational Therapy Students' Perceptions of Learning to Coach" was published in 2022. Journal: Occup Ther Int.

### 1.2. Occupational Therapy Coaching Models

Within OT, different ICF-related coaching models have been developed, including solution-focused coaching, occupational performance coaching, occupation-based coaching, and coaching in context (CinC) [3, 4, 20, 22–24]. Regardless of the model, when an ICF coaching lens is used in OT practice, clients set their own priorities, which become the goals directly addressed during sessions [6, 19, 21, 22]. Further, OT coaches approach clients with an interest to truly bring forth their lived experience, empower them to utilize their own insights to find novel solutions or adapt strategies, and develop action plans to achieve their goals [4, 6, 20]. Coaching capitalizes on client motivation and resourcefulness rather than using a clinician-expert approach [21, 22]. These essential and unique actions of OT coaches also emerged in a coaching fidelity study [5]. These same authors identified behaviors used in other OT approaches that are not compatible with coaching, such as focusing on skills in isolation, choosing activities for the client, making recommendations, and giving a “home” program [5]. Coaching in context (CinC) is an OT-developed coaching model that possesses all the ICF-style coaching characteristics. The CinC model was the approach taught to OT student participants in the study described in this article.

### 1.3. Coaching in Context Model

The CinC model is adaptable to any occupation, setting, or population and has been found effective with college students with disabilities [3, 22], adults with spinal cord injuries [4], caregivers of people with strokes [25], and informal care partners of children with spinal cord injuries., [9]. This model was developed as an interprofessional approach that operationalizes ICF competencies into three components, *Connect*, *Discover*, and *Plan*, and five distinct attributes: active listening, reflective responding, skillful questioning, grounded in context, and leveraging strengths [11]; Coronado et al., 2022; [22, 25, 26]. The components are the framework, whereas the attributes are the behaviors that permeate the coaching session (Coronado et al., 2022). The *Connect* component has the dual purpose of cultivating the relationship between client and coach and establishing the goal of the coaching session [11]; Coronado et al., 2022. The *Discover* component is a space where clients can explore their strengths, gain insights into their own occupational performance, and identify potential solutions that they can then leverage to achieve their goal(s) [11]; Coronado et al., 2022. During the *Plan* component, the client identifies strategies that will allow them to make progress toward their goals, formulates these strategies into a concrete action plan, and identifies potential pitfalls to this plan [11]; Coronado et al., 2022.

The article "“I Could Really Use This”: Occupational Therapy Students' Perceptions of Learning to Coach" was published in 2022. Journal: Occup Ther Int.

### 1.4. Occupational Therapists' Perception of Coaching

Coaching is not typically taught with entry-level OT education [11]; however, OT practitioners have acquired these skills through professional coaching schools, OT-specific professional development courses, and rehabilitation-focused coaching courses. Four studies to date have explored the perceptions of experienced rehabilitation professionals, including occupational therapists, about the value of incorporating coaching within their practice [6, 10, 12, 27]. The rehabilitation professionals reported improved flexibility, listening skills, collaboration, and goal development [6, 27]. They noted a shift in their mindset from the therapist as the expert to the therapist as the facilitator of change, which was freeing [6, 27]. They perceived that coaching resulted in clients finding solutions for their own goals [10]. They also reported an increased ability to empower and engage their clients [6]. Further, they perceived that their coaching clients took ownership of their own choices [6, 12]. This led these practitioners to have an enhanced perception of their own effectiveness [6, 12].

Coaching requires skills that expand upon what OT students learn in current academic curricula and what occupational therapists use in their day-to-day practice.

In-depth training in coaching is needed before practitioners can effectively integrate this approach into their practice [6, 10]. Incorporating coaching into OT students' educational experience may allow them to develop these skills prior to independent practice. However, it is unclear if OT students, as novice practitioners who are still forming their professional identity and skills, would see the same value in learning to coach as experienced practitioners.

The article "“I Could Really Use This”: Occupational Therapy Students' Perceptions of Learning to Coach" was published in 2022. Journal: Occup Ther Int.

### 1.5. Rationale and Objectives

This study is aimed at providing insight into OT students' occupational experience with learning coaching while completing their entry-level education, specifically their Level II fieldwork.

A phenomenological study was conducted with the objectives of exploring OT students' perceptions of (1) the benefits and challenges of learning coaching while in fieldwork, (2) the value of developing coaching skills for their future OT career, (3) how applicable coaching is to other OT practice settings, and (4) the benefits experienced by the OT clients.

## 2. Materials and Methods

### 2.1. Participants

All OT students (*n* = 14) who completed their Level II fieldwork within the GOALS^2^ Program from 2017 to 2020 received in-person invitations and chose to participate in the study. The university institutional review board approved the study, and all participants signed written consent forms after engaging in an informed consent process. The OT students were made aware that choosing to participate in the study had no impact on their fieldwork placement. Participants' sociodemographic information was collected via self-report and is summarized in Table 1. Of all participants, 13 identified as women, as expected given that most occupational therapists in the United States are women. The mean age of the participants was 30.6 years (SD = 7.6), and for seven participants, OT was not their first career.

### 2.2. Research Team

The research team was composed of five authors, and their work was supported by several graduate assistants. All members of the research team self-identified as female and white; two self-identified their ethnicity as Hispanic/Latina. All members were occupational therapists (1st author) or OT students. The first author has extensive experience in qualitative and quantitative research methodology. Authors 2-5 were entry-level occupational therapy doctoral students completing this work as part of their capstone project at the time of the study; they were novices in qualitative research. The 1st author is a full-time faculty member in an OT program, the administrator of the GOALS^2^ Program, and one of two people who provide coaching training to the Level II fieldwork students placed with the program. Additionally, she served as the primary instructor for four courses in the didactic portion of the Level II students' academic program. To minimize the potential effect of the 1st author's multiple roles with the participants, the informed consent process was completed by the graduate assistants. Similarly, the 1st author participated in the data analysis at the refinement stage of the coding matrix and theme identification but did not have firsthand involvement with data collection and initial data analysis of the study methodology. Authors 2-5 completed their doctoral experiential and capstone project within the GOALS^2^ Program during the two academic years that followed data collection for this study. The roles of the graduate assistants and the training they received are described in Data Collection and Data Analysis. All members of the research team were trained in coaching and had used coaching within OT practice.

The article "“I Could Really Use This”: Occupational Therapy Students' Perceptions of Learning to Coach" was published in 2022. Journal: Occup Ther Int.

### 2.3. Setting

The GOALS^2^ Program is a Level II fieldwork placement that offers OT services using the ICF-style coaching approach CinC to university students who have disabilities [3], [22]. The OT students who completed, in pairs, a Level II fieldwork with the GOALS^2^ Program were trained in CinC over the 12 weeks of their placement under the instruction and supervision of licensed occupational therapists who are certified coaches. The training included two 3-hour introductory trainings to coaching and CinC via practicing skills, weekly discussions of coaching-related topics, readings, role modeling from experienced OT coaches, supervised OT-coaching sessions, and weekly case reviews with feedback of videos of coaching sessions. A distance supervision model was used with the primary preceptor on site 8-12 hours per week and a secondary preceptor available as needed. The primary preceptor had been an occupational therapist for 4 years at the beginning of the study and was new to Level II fieldwork preceptorship. These OT students are uniquely situated to provide insights into the value of learning and using coaching while becoming occupational therapists.

The OT fieldwork students with the GOALS^2^ Program who became participants in this study completed the didactic portion of their OT education in one of three programs within one university. The participants had received minimal coaching training as part of the didactic portion of their OT educational program. Some of the participants had received a two-hour lecture and laboratory experience within a course, whereas others had heard of coaching briefly in coursework.

### 2.4. Data Collection

The data for this phenomenological study were collected through audio-recorded semistructured interviews that took place within two weeks of the end of each participant's 12-week fieldwork experience. The interviews were conducted by trained graduate assistants using an interview guide that included a series of open-ended questions and follow-up probing questions. The interview questions focused on the participants' experience within this fieldwork without asking specifically about coaching to minimize the risk of biasing their answers (Table 2). Interviews were conducted one-on-one, either in person or through distance meeting technology at a time that was convenient to participants. Each participant was interviewed once, and the interviews ranged from 20 to 60 minutes depending on the depth of information shared by participants.

The article "“I Could Really Use This”: Occupational Therapy Students' Perceptions of Learning to Coach" was published in 2022. Journal: Occup Ther Int.

### 2.5. Data Analysis

A multistep, iterative process including preparing the data, developing the codebook, coding, and data interpretation was used as described below.

*Data Preparation and Code Book Development*. To prepare the data for analysis, all interviews were transcribed verbatim using a transcription protocol, checked for accuracy by a 2nd transcriber, and deidentified by trained graduate assistants. An inductive approach was utilized to develop the codebook using an iterative multicoder process. This process included reading interview transcripts to identify codes, writing and refining codes' definitions, creating and adjusting codes' hierarchies, and consulting with a senior researcher. This process was conducted by two researchers (author 2 and author 3) with guidance and input from a senior researcher (author 1). An audit trail and reflexive journals were maintained throughout this process and the data analysis more broadly.

*Coding*. Once the codebook was finalized, all transcripts were uploaded into NVivo (Version 12). Two of the researchers (author 2 and author 3) coded all 14 transcripts independently. These researchers then compared their coding to identify differences, and all differences were resolved through discussion. Intercoder reliability for each transcript was consistently above ~95% agreement. Saturation was achieved, as no new insights or understandings emerged beyond the codes included in the codebook.

*Interpretation*. With all interviews coded, themes were identified from that data using a nonlinear, phenomenological, and narrative inquiry process, in which two of the researchers (author 2 and author 3) independently examined the data organized by codes to illuminate themes. This was followed by peer debriefing between the two researchers to examine areas of agreement or disagreement and gain a deeper understanding of what the data was revealing [28]. The researchers reviewed their audit trails and reflexive journals to ensure that their interpretation had not missed key elements. Expert debriefing with the senior author (author 1) occurred to confirm the rigor and interpretation of the analysis [28]. Interpretation of data was confirmed via member checking with current and former Level II OT fieldwork students who participated in the GOALS^2^ Program.

The article "“I Could Really Use This”: Occupational Therapy Students' Perceptions of Learning to Coach" was published in 2022. Journal: Occup Ther Int.

## 3. Results

Three themes emerged from the data analysis process: *Coaching Requires a Mindset Shift*, *Change is a Journey*, and *Impact on Clients.* These themes and their eight subthemes are listed in Figure 1 and explicated with examples in the following paragraphs.

### 3.1. Coaching Requires a Mindset Shift

Most participants commented on coaching demanding a shift in mindset from more traditional OT practice. One participant captured this idea when stating that coaching required them, as novice practitioners, to change their “way of thinking” (Participant 11 [P11], Line 119-120 [L119-120]). Three subthemes emerged from the data characterizing this mindset shift: *Reimagining of Roles*, *Flexibility*, and *Time*.

#### 3.1.1. Reimagining of Roles

The OT practitioner is often cast in the role of an expert who, through the OT process, helps the client reach goals that are meaningful to them [3, 19]. In contrast, one participant described coaching as “facilitating client success through the development of their own goals, achieving their own independence … and coming up with [strategies and plans] themselves” (P6, L178-180). This mindset shift required a reimagining of roles for the participants. However, accepting that clients have expertise was difficult for some participants, such as the participant who noted learning to coach “can be overwhelming [at first] to people that aren't familiar with it” (P11, L119-120) and another who stated they wanted to “jump in and be the expert” (P14, L142-143) and that “not being able to [be the expert] can be one of the more challenging components of coaching” (P14, L142-143). Another participant noted that this shift was often more difficult for the OT coach than the client, stating “I think it's more frustrating for the practitioners because we felt like we're not able to help [them] make progress” (P11, L193-194). On the other hand, participants realized that this assumption about practitioners being the sole expert in the practitioner-client relationship is false. This is best captured by a participant who stated “we're not the expert. People really do have the knowledge, and they know themselves the best” (P12, L69-71). This reimagining of roles was not only for the OT coach. Participants noticed that clients were experiencing this shift; one participant stated, “giving people an opportunity to say what's on their mind is important, and both clinicians and clients aren't always the most comfortable with [that],” adding that “[some] clients come in thinking [the clinician is] the expert, [that they] should have all the answers” (P8, L98-102). Another participant explained, “the client comes back every week, and checks in, and says ‘oh, this strategy didn't quite work. Let's rework it a little bit.' So, it's … really, really interesting to see them problem-solve rather than us just doing it for them” (P14, L114-117). This reimagining of roles takes time and is in part related to noticing positive impacts on clients.

The article "“I Could Really Use This”: Occupational Therapy Students' Perceptions of Learning to Coach" was published in 2022. Journal: Occup Ther Int.

#### 3.1.2. Time

All 14 participants mentioned “time” during their interview, specifically the time afforded for coaching and the value of giving clients time to change. Participants noted that the ability to schedule sessions for the duration that each client needed enhanced their ability to fully engage in the coaching process. Participant Three remarked, “if [a client] needs 2 hours, you can give them 2 hours. If they only need 45 minutes, that's fine too” (L215-216). While a coaching session can be effectively completed in as little as 20 minutes, participants noted the additive value of multiple coaching sessions on clients. One participant stated, “the [coaching] process builds on itself” (P14, L114-117). Another participant described how they “needed to get more comfortable with [progress] taking a longer time than I expected. Sometimes you just need to plant the seed in somebody's mind” (P5, L149-154).

#### 3.1.3. Flexibility

Participants remarked on needing to be adaptable when working with clients using a coaching approach. This adaptability took many forms and went beyond what they would have typically experienced as occupational therapists. One participant stated, “I love the flexibility of [coaching]. I think that this [flexibility] benefits the clients” (P3, L252-253). In coaching, flexibility is in part related to adapting to clients' shifting priorities. The OT coaches work on what is important to the client at that moment. For example, one participant recalled that “clients can come in crisis modes. [They have] emergencies, projects, or something that's weighing heavy on them and takes the focus away from their [long-term] goals” and the need in these instances to “embrace [the fact] that things were unpredictable,” (P14, L323-328) and “to adjust strategies, [for example] how I paced my questioning” (P1, L166-172). One participant reflected, “the coaching model helps us as occupational therapists [to] meet people where they are” adding “coaches [don't] project [their thoughts] on the situation, [they simply] work with them” (P8, L132-136).

### 3.2. Change Is a Journey

Participants remarked on the development of their own coaching skills and clients' progression toward change. One way that participants conceptualized this transformation within the coaching model was employing language from the Transtheoretical Model of Change: “understanding where each client was in their journey to change” ([29]; P10, L71-72). For example, “if the client was [in] precontemplation, they knew they were experiencing challenges on campus, but they couldn't exactly identify it, or they weren't ready to make steps toward the change. [Then,] it was a little more challenging during the sessions” (P10, L76-78). This understanding of their clients' journey to change allowed participants to hone their own professional reasoning and develop reasonable expectations of clients. One participant remarked, “you think that just in one session you're supposed to solve everything, but the way that [coaching] actually works is that you chip away at things slowly, be patient, and wait for [progress] to happen” (P5, L151-154). Three subthemes emerged related to *Change is a Journey*: *Motivation is Key*, *Developing Skills and Confidence*, and *Therapeutic Relationships.*

The article "“I Could Really Use This”: Occupational Therapy Students' Perceptions of Learning to Coach" was published in 2022. Journal: Occup Ther Int.

#### 3.2.1. Motivation Is Key

Coaching gave participants the opportunity to develop their ability to explore their client's motivation for change, which they saw as generalizable to future practice settings. Participant Ten opined, “I think that coaching really helps to dig into [clients'] values [and] as to why participating in OT coaching is important” (L282-283). Developing an understanding of their client's patterns of behavior was a crucial element of enacting change. One participant noted that “it's about trying to peel back the layers and get to why they are doing what they're doing or not doing… Until you can get to that, there really isn't going to be much change” (P3, L134-136). Taking a deep dive to better understand client motivation and participation was a coaching skill that participants, as novice practitioners, noted had the potential to enrich their future OT practice, regardless of the setting. One participant explained, “The traditional [OT] model is to label clients who aren't following recommendations as non-compliant. [Through coaching you realize that] it is not the case. It's probably that they're not [motivated] about the plan, [unsure] how to implement it, [or] confused by the directions” (P10, L295-297). Another participant reflected, “[I'm] going to take that idea of figuring out what my client's end goal is,… their motivation,… [and] why they want to be in therapy … into more traditional OT settings” (P14, L298-303).

#### 3.2.2. Developing Skills and Confidence

Participants reflected on their journey of developing coaching skills and professional reasoning through the process of coaching clients. One participant asserted, “[through] my experience over the course of the semester, I've evolved as I've continued to work with clients” (P1, L289-290). One participant explained that coaching enables them to enact core OT principles when explaining that professors “talk about [being client-centered] the whole time we've been in school … [but] that's easier said than practiced. I am going to have a much stronger ability to be client-centered now [after learning to coach]” (P11, L369-374). When describing the skills and confidence they built, participants noted the following areas of improvement: “[client] interaction, interviewing [and] being comfortable but professional” (P3, L188); “therapeutic use of self, clinical reasoning, active listening, [and] being able to really understand what my client needs, meet them where they're at, and support them” (P14, L65-68); “getting the full story” from clients (P9, L96-97); “slowing down instead of jumping right in and trying to fix” (P10, L465-466); “learning what I can do as an occupational therapist outside of typical [practice]” (P4, L69-72); and “confidence establishing relationships with clients” (P2, L444-445). Many of these skills are related to therapeutic relationships and thus directly applicable to more traditional OT practice.

The article "“I Could Really Use This”: Occupational Therapy Students' Perceptions of Learning to Coach" was published in 2022. Journal: Occup Ther Int.

#### 3.2.3. Therapeutic Relationships

As participants reflected on the knowledge they gained through learning about coaching, the importance of therapeutic relationships emerged. Participant Twelve explained, “I think that the foundation of any type of therapeutic work is to be able to build that relationship” (L117-119). Participants reported that building a therapeutic relationship is essential to coaching. One participant remarked, “the coaching process is all about discussion, connection, rapport building, and therapeutic use of self” (P7, L107-108). Building this collaborative relationship allowed for greater insight into clients and improved professional reasoning on the part of the fieldwork student. One participant stated that the client-practitioner relationship allowed them to understand “what exactly [clients were] trying to get out of the GOALS^2^ Program,… clients' different needs, and different things that would help them to succeed” (P13, L124-126). Participant Twelve emphasized that trust is vital to the therapeutic relationship alongside technical skills as a practitioner, asserting, “if you cannot build relationships with people, [even if you are otherwise] the most skilled practitioner in the world, [clients won't] trust you. They're not going to want to work with you” (L153-156). Thus, developing a therapeutic relationship is a skill critical to coaching that is transferable to other areas of practice. Therapeutic relationships led to client open-mindedness and enjoyment of OT-led coaching sessions. One participant stated, “if you build this connection with a client, then they're more willing to be open to you. GOALS^2^ Program clients were really excited to come back to their sessions” (P13, L160-165).

The article "“I Could Really Use This”: Occupational Therapy Students' Perceptions of Learning to Coach" was published in 2022. Journal: Occup Ther Int.

### 3.3. Impact on Clients

Client impact was inextricably linked to participants' assessment of their own skill development and implementation of coaching. Every participant mentioned the effect they perceived they had on clients through coaching. One participant noted that clients developed self-confidence while working toward their goals, observing “how much confidence people could build by coming up with solutions for themselves” (P11, L86-87). Another participant stated that clients would say things such as “‘wow, I thought of that on my own'” (P11, L88-90), which was empowering for clients.

The positive impact of the coaching model shifted the dynamic of the session, which became evident when participants moved away from the client-led approach and became increasingly directive. For example, participant Five recalled, “throughout the semester, we were working on what [clients] wanted to work on, but if at any point that changed and we started acting in a more directive way, you could see the client become a little less interested” (L197-202). All these skills increased follow-through and improved outcomes for clients. As one participant stated, “[coaching] helps with [client] outcomes because people are more invested, and it's actually a solution that [is] achievable for them. And I don't know that I would have seen it quite that way if I hadn't [learned to coach]” (P11, L379-390). Two subthemes emerged from this larger theme of the impact on clients: *When it Works, it Works!* and *Is Coaching for Everyone?*

#### 3.3.1. When It Works, It Works!

One participant captured this theme when stating, “it's magic” (P7, L427-429). [Clients] “know what their issues are, by and large” (P7, L427-429). Participant Fourteen found that brainstorming was the most helpful, asserting, “brainstorming especially was where I saw the biggest shift in our clients and the most progress” (L173-180). Participants “tried the strategies” (P7, L427-429; P14, L173) on their own and “modified them throughout the week” (P14, L173-180). The coaching process also promotes long-term independence; one participant stated, “we've given [clients] tools to do it on their own. That's our goal, to support them now [so] they can transfer those skills later” (P3, L289-291). Overall, the Level II OT fieldwork students found that coaching helped clients, but coaching is not necessarily for everyone.

The article "“I Could Really Use This”: Occupational Therapy Students' Perceptions of Learning to Coach" was published in 2022. Journal: Occup Ther Int.

#### 3.3.2. Is Coaching for Everyone?

Participants in this study noted that some clients had trouble with the coaching process. For some, the difficulty was perceived to be grounded in motivation. One participant asserted, “coaching really only works if there's some self-motivation in the client” (P6, L23-24). However, motivation can be fostered in clients; it is not an impasse. This was illustrated by a participant who stated, “[Clients] would come up with a strategy, and [I would ask] ‘Are you going to try it?' [The] clients would admit ‘No, because I'm not really motivated.' [We] researched how to help them find motivation” (P10, L60-65). For other clients, the challenge was the conversation-based nature of the coaching approach. Participants recalled a client who “had been coming to the program and participating for a long time, but it was hard to make a connection and follow the process with him because there just wasn't a whole lot of back and forth [conversation]” (P7, L161-163). The participants needed to adapt the coaching process given the clients they were serving, some of which had difficulty communicating and engaging in abstract conversations. Finally, the client's ability to self-reflect is key to success in coaching. One participant assessed, “the coaching model was really challenging [with some clients] because sometimes that ability to reflect deeply or think of creative new ways to do things was really a challenge [for the client]” (P11, L129-130). Although coaching works for many, adapting the coaching model or considering other approaches is necessary for some clients. Coaching is only one tool in an occupational therapist's toolbox.

## 4. Discussion

This study aimed to explore OT students' perceptions of learning and using the CinC model while completing Level II fieldwork. While ICF-style coaching has a large body of evidence in other fields, it is relatively new within the OT profession [2]. Most occupational therapists do not learn coaching skills during their entry-level education [6]. A few studies have explored the perspective of licensed occupational therapists introducing coaching into their practice [6, 12, 27], but there is no research on students' perceptions of learning this approach within OT education. Overall, OT students who participated in this study found value in learning and using coaching as an approach to address clients' goals, with three themes emerging from the analysis.

Coaching requiring a “mindset shift,” even for novice practitioners, permeated the data. In the view of participants, coaching allowed for a more collaborative and flexible approach compared to traditional OT practice by shifting the power dynamic that exists between clients and practitioners toward the empowerment of clients. As found in previous studies, the coaching relationship emphasized the expertise of the client in their own life and the expertise of the coach as the facilitator of problem-solving and self-efficacy for the client [6, 19] as they work toward “achieving their own independence … and coming up with [strategies and plans] themselves” (P6, L178-180). The concept of coaching requiring a *Mindset Shift* is consistent with prior research with licensed practitioners who remarked that implementing coaching fostered a positive change in their practice [6, 12]. By dissolving the perception that the occupational therapist is the expert [6], the client and OT coach can develop strategies to address occupational challenges more effectively, as clients “really do have the knowledge, and they know themselves the best” (P12, L69-71).

The article "“I Could Really Use This”: Occupational Therapy Students' Perceptions of Learning to Coach" was published in 2022. Journal: Occup Ther Int.

Within this study, participants experienced a shift in perspective from therapist-expert to client-expert and identified this shift as a difference between traditional OT and OT-led coaching. Consistent with the participants' perspectives, experienced occupational therapists noted in previous studies that they had to change their role from expert to facilitator and that preventing oneself from intervening as an expert was difficult [6]. This shift allowed clients to create relevant and meaningful goals and allowed the OT coach to adjust priorities and share only targeted information with the client as needed while emphasizing the client's personal problem-solving skills [19, 30]. Using a coaching model to guide sessions, occupational therapists noted that they increased their flexibility to remain client-centered in their approach [6, 30]. OT students in this study explained the value of conducting coaching sessions in a way that was adaptable to client needs, ranging from adjusting the duration and frequency of sessions to alternating between areas of focus throughout and even within sessions. These same students reflected on adjusting their therapeutic use of self, taking client context into consideration, and letting go of judgment or personal investment, all of which allowed clients to shift their mindset, embrace their knowledge and power, and strive toward their goals, as found in previous studies [4, 22]. In one study, clients expressed feeling supported in the open environment of OT-led coaching, which they perceived led to their academic and personal growth [22].

OT students in this study and experienced occupational therapists in previous studies grounded their evaluation of the coaching process on the effect it had on clients [6]. Participants in this study emphasized that coaching is a means to achievable, sustainable solutions developed by clients, while licensed occupational therapists placed greater emphasis on coaching as a process for effective and clear goal development [6]. Both expressed coaching as a confidence-building intervention for clients and discussed moments when coaching fell into place [6]. Participants in this study emphasized the long-term implications of confidence, insight, and techniques that clients can apply outside of coaching sessions. However, they also discussed client factors that made coaching difficult for some clients with disabilities. They noted factors such as low motivation, communication skill challenges, and inability to self-reflect as barriers. OT practitioners in a previous study, however, emphasized their own biases as a barrier to coaching, specifically managing conflicting opinions regarding the ethics of client decision-making [6]. The role of the practitioner as a coach is to take on the client's views, withhold judgment, and gently invite them to explore novel strategies or solutions of their own creation [4, 6]. With a coaching mindset, the OT students who participated in this study believed that occupational therapists can more deeply cultivate a therapeutic relationship using coaching across practice settings.

The article "“I Could Really Use This”: Occupational Therapy Students' Perceptions of Learning to Coach" was published in 2022. Journal: Occup Ther Int.

Participants in this study remarked on coaching as a means of improving practitioner competency and confidence, in addition to increasing clients' personal insights. Student practitioners placed emphasis on the therapeutic relationship as the foundation of any productive clinical interaction and a means to client involvement and success, applicable to any practice setting. This is consistent with experienced occupational therapists who noted that the rapport built via coaching, by improving listening skills, engendered greater disclosure from clients [6]. Other study findings emphasized the perceptions of coaching service providers, stating that their skilled interactions and observations of clients have a direct impact on actively facilitating and enhancing a client's state of engagement, motivation, and real-life outcomes [12]. Experienced occupational therapists in previous studies focused less on skill building and developing confidence as practitioners but still noted that coaching increased their own perception of effectiveness [6]. For occupational therapists, increased effectiveness was linked to embracing client expertise and liberating themselves from a “fixing” role [6].

### 4.1. Implications

Overall, the participants in this study valued learning coaching in their Level II fieldwork; they saw a congruency between coaching and core OT principles. Learning to coach, in their view, equipped them with skills to more fully enact core OT principles, such as client-centered care and therapeutic use of self. They perceived that the value of learning to coach within this setting would benefit them in any other practice setting. This study adds to the fast-growing body of evidence about the value of coaching within OT practice. This evidence suggests that incorporating coaching into the OT curriculum would be advantageous, as students would learn coaching skills early in their careers and could apply those coaching principles to improve future client outcomes. Thus, entry-level OT educational programs should explore ways to incorporate coaching training within their curriculum. OT practitioners are encouraged to seek continuing education opportunities in which they can learn to infuse ICF-style coaching within their own practice. Knowledge translation takes time; however, organizations such as the American Occupational Therapy Association and the World Federation of Occupational Therapy play key roles in fostering changes in OT practice when new research evidence emerges.

The article "“I Could Really Use This”: Occupational Therapy Students' Perceptions of Learning to Coach" was published in 2022. Journal: Occup Ther Int.

### 4.2. Limitations

Although the sample size (*n* = 14) was appropriate for a qualitative study, the transferability of the study results is limited given that all participants completed their fieldwork within the same role-emerging fieldwork site. While efforts were made throughout the study to minimize research bias (i.e., reflexive journaling, audit trail, multiple coders and independent thematic analysis, member checking, and peer debriefing with a senior researcher), as in all qualitative studies, there is still the possibility of research bias within the results. Interviews, as a data source, rely on participants' subjective experiences, which are not an objective indicator of a participant's growth in skills. The results are also limited by the participants' own ability to self-reflect.

### 4.3. Future Directions

Duplication of this study with participants from various fieldwork sites would help differentiate between the coaching and site-specific experiences of participants. Further, exploring the value of teaching coaching within the didactic portion of the program could be explored. Another logical next step would be to explore the degree to which coaching principles learned in fieldwork are utilized by licensed occupational therapists once practicing in a variety of settings. Finally, studies exploring the characteristics of individuals and the context in which coaching is less efficacious are needed.

The article "“I Could Really Use This”: Occupational Therapy Students' Perceptions of Learning to Coach" was published in 2022. Journal: Occup Ther Int.

## 5. Conclusions

Coaching requires a different skill set than what most occupational therapists traditionally learn in academia and use in their day-to-day practice. Level II OT fieldwork students perceived coaching as a useful approach that improved their therapeutic relationships, skills, flexibility, and confidence. Moreover, coaching allowed students to empower clients to be experts, explore clients' contexts, and develop professional and realistic expectations of client change. Participants discussed the coaching concepts and skills they utilized in this Level II fieldwork as beneficial for clients, including individuals whom they will work with in future practice. Coaching was characterized as a valuable intervention to execute concepts taught within the OT curriculum, such as emphasizing client-centered care and initiating a shift away from a practitioner-directed model toward a more effective model that emphasizes greater client autonomy.

## Figures and Tables

**Figure 1:** Themes and subthemes related to Level II OT fieldwork students' perceptions of coaching.

**Table 1:** Study participants' sociodemographic information.

Characteristics	Frequency (*n*)	Percentage (%)
*Gender identity* ^a^		
Woman	13	92.9
Man	1	7.1
*Age (years)*		
20-24	4	28.6
25-29	4	28.6
30-34	2	14.3
35-39	2	14.3
40-44	1	7.1
45-49	1	7.1
*Ethnicity/race* ^b^		
White		
Black or African American, Hispanic or Latino, native	13	92.9
American, Asian	1	7.1
*Program being completed while in Level II fieldwork*		
MSOT	12	85.7
OTD	2	14.3
*Highest degree held prior to beginning OT program*		
Bachelor's degree	13	92.9
Master's degree	1	7.1
*Nontraditional student/2^nd^ career student*		
Yes	7	50
No	7	50

Notes. MSOT = Master of Occupational Therapy; OTD = Occupational Therapy Doctorate; ^a^participants were asked to write their gender identity; ^b^participants were asked to write their ethnicity/race.

**Table 2:** Sample semistructured interview questions.

(i) Tell me about 1-2 experiences from this fieldwork, if there was any, that had particular meaning or influence on you as a future occupational therapist
(ii) What would you tell future fieldwork students about the value of this fieldwork experience for their learning?
(iii) What do you think will be the impact of this fieldwork on your future practice?

## Data Availability

The data used to support the findings of this study are available from the corresponding author upon reasonable request.
